# Multisemantic Level Patch Merger Vision Transformer for Diagnosis of Pneumonia

**DOI:** 10.1155/2022/7852958

**Published:** 2022-06-21

**Authors:** Zheng Jiang, Liang Chen

**Affiliations:** Department of Radiology, The First Affiliated Hospital of Chongqing Medical University, 400016, China

## Abstract

The most popular test for pneumonia, a serious health threat to children, is chest X-ray imaging. However, the diagnosis of pneumonia relies on the expertise of experienced radiologists, and the scarcity of medical resources has forced us to conduct research on CAD (computer-aided diagnosis). In this study, we propose MP-ViT, the Multisemantic Level Patch Merger Vision Transformer, to achieve automatic diagnosis of pneumonia in chest X-ray images. We introduce Patch Merger to reduce the computational cost of ViT. Meanwhile, the intermediate results calculated by Patch Merger participate in the final classification in a concise way, so as to make full use of the intermediate information of the high-level semantic space to learn from local to overall and to avoid information loss caused by Patch Merger. We conducted experiments on a dataset with 3,883 chest X-ray images described as pneumonia and 1,349 images labeled as normal, and the results show that even without pretraining ViT on a large dataset, our model can achieve the accuracy of 0.91, the precision of 0.92, the recall of 0.89, and the *F*1-score of 0.90, which is better than Patch Merger on a small dataset. The model can provide CAD for physicians and improve diagnostic reliability.

## 1. Introduction

Pneumonia is an infectious inflammation of the alveoli, distal airways, and interstitial spaces of the lungs and is mainly triggered by bacteria and viruses. It is the number one killer of children under 5 years old and poses a major threat to children's health, causing more deaths than malaria, tuberculosis, and AIDS combined [1–3]. The World Health Organization (WHO, Geneva) states that childhood pneumonia leads to approximately 1.4 million deaths per year, accounting for about 18% of deaths among children under 5 years old worldwide [4]. This has prompted an increasing interest in fast and low-cost pneumonia detection means.

There are many common tests for pneumonia in children, such as chest X-ray, chest computerized tomography (CT), and magnetic resonance imaging (MRI). Although less accurate than CT and MRI, X-ray is the cheapest, the most easily accessible and the most needed examination for developing countries, where medical resources are relatively in short supply [5, 6]. The correct diagnosis by chest X-ray depends on the knowledge of experienced physicians, who are also scarce in developing countries. Therefore, how to help physicians improve diagnosis accuracy by computer-aided diagnosis (CAD) technology is a meaningful topic.

Deep learning technology can be used to provide CAD and improve the accuracy and efficiency of clinical diagnosis. It automatically extracts features layer by layer from the raw data and finally builds mathematical models. Those models that have achieved advantages in various competitions (such as ImageNet Large-Scale Visual Recognition Challenge (ILSVRC) [7]) in the field of computer vision (CV) are applied on medical images to provide advice on diagnosis.

In 2012, Krizhevsky et al. [8] used convolutional neural network (CNN) and achieved overwhelming success in the ImageNet challenge, which attracts extensive research attention. After the success of CNN models [8–10], the literature [11] used CNN to analyze medical images; the literature [12] used CNN-based EfficientNet to train a classifier by transfer learning and fine-tuning for diagnosis of pneumonia. In 2020, Dosovitskiy et al. proposed the Vision Transformer (ViT) model [13], which achieves comparable or even better classification performance than CNN with lower computational cost, making ViT model a hot research topic in CV field. Some studies have tried to apply it on the medical image tasks, e.g., comparing the performance between ViT and some other models and proposing to use ViT for pneumonia diagnosis [14], or improving ViT for COVID-19 detection [15]. To reduce the computational efforts of ViT, in 2022, Renggli et al. [16] proposed the Patch Merger, which significantly reduces the computational efforts of ViT while maintaining the model performance basically unchanged. However, there are some risks in applying Patch Merger, because some patches containing important information may be discarded during merging, which may be a problem especially for medical image datasets.

Inspired by that work, we propose the Multisemantic Level Patch Merger Vision Transformer (MP-ViT). It moves the Patch Merger Block forward and preserves the intermediate results participated in the final classification.

The main contributions of this study are listed as below:

1. We proposed the Patch Fuser, a concise method for memorizing and utilizing intermediate information in the semantic transformation process of the Patch Merger model, thus, making full use of feature information in the semantic space of different levels
2. We further reduced the computational efforts of ViT by moving the Patch Merger Block forward, while keeping the classification performance of the model
3. Through experiments, we showed that MP-ViT can maintain the advantages of Patch Merger, while avoiding the risk of losing the higher-level semantic information in Patch Merger

The structure of the body in this paper is as follows.

In Related Work, we briefly reviewed the related researches on Transformer, ViT, and Patch Merger and introduced their applications in CV and medical imaging tasks. Meanwhile, the deficiencies and risks of these models were also raised.

In Methods, we described the principles and structures of Transformer, ViT, and Patch Merger and detailed our Patch Fuser and MP-ViT models that have been proposed, as well as the label smoothing technique.

In Experiments, we introduced the dataset, the image enhancement method, and our experimental details. We compared the performance of those models together with ResNet50, which played the role of baseline, and showed that our model has won the best performance in the experiment. We analyzed these models while taking comparison between them.

In Conclusion and Future Work, we summarized the advantages of our proposed model and also analyzed the shortcomings of our current work while proposing the next step of future research work.

## 2. Related Work

Medical imaging technology has made tremendous progress in the past few decades. Traditional machine learning methods for solving medical imaging tasks mainly rely on the expertise of medical experts to carry out mathematical modeling [17], but these methods cannot take full advantage of the expressive power of large image datasets and have not yet met the requirements for doctors to improve diagnostic accuracy and workflow efficiency. As deep learning has become the state-of-the-art machine learning approach, especially after the overwhelming victory of CNN in CV competitions, there have been more and more cases using deep learning methods to analyze medical images, such as classification tasks to distinguish normal and diseased tissues, benign and malignant tumors, and image segmentation tasks to extract the boundaries of normal or diseased tissues or organs to obtain normal or diseased regions [18–20]. However, these cases have not yet fully analyzed and exploited the relationship of pixels at long distances on the image. The costs are also quite expensive.

The Transformer model [21] originated in the field of Natural Language Processing (NLP), which avoids model architectures of recursion and CNN and completely relies on attention mechanisms to obtain global dependencies between inputs and outputs. This architecture significantly increases parallelization level, thus achieving better translation quality while substantially improving the speed of computation. Once proposed, it quickly dominated the NLP field.

Based on the Transformer's success in field of NLP, the CV community has also tried to assimilate Transformer's ideas by integrating attention mechanisms [21–23] into CNN-like architectures [24, 25], which either applies attention with CNN or replaces some certain architectures of CNN with attention. Cordonnier et al. [26] proposed to apply a complete self-attentive mechanism in 2 × 2 image patches. In 2020, Dosovitskiy et al. [13] argued that applying the attention mechanism while maintaining the overall architecture of CNN is unnecessary and that the Transformer model can be applied directly to the sequence of image patches segmented from the original image, thus, completely replacing the standard convolution in deep neural networks, and proposed the Vision Transformer model. Since its proposal, the ViT has shown to be the most advanced model in many tasks in CV. In addition to the aforementioned image classification task, for object detection, Zhu et al. [27] proposed Deformable Transformer (DETR), which improves the self-attention mechanism of ViT by focusing only on a small number of critical samples near the reference point. In the field of semantic segmentation, Zheng et al. [28] replaced the convolutional network with a pure Transformer to build Segmentation Transformer (SETR), which achieved better performance than CNN approaches. In the area of image colorization, Kumar et al. [29] used a conditional autoregressive axial transformer to implement the coarse colorization of grayscale images at low resolution, which was proved to achieve better results than previous means with lower computational complexity. In low-level CV tasks (e.g., denoising, superresolution, and deduplication), instead of directly slicing the original image into patches, Chen et al. [30] first fed the image to a specific header, then segmented the generated features into small patches that were passed to Transformer, and finally developed a pretrained model, whose performance is better than that of all models before Transformer's advent by utilizing Transformer's powerful representation capabilities on large-scale datasets. In the video understanding task, Arnab et al. [31] used several Transformer layers to process the time-spacial markers extracted from the input video and resolved the problem of long time-spacial marker input sequences through several different methods and achieved the state-of-the-art results on five popular video datasets. Matsoukas et al. [32] collected three medical imaging datasets and compared the classification performance of CNN and ViT with different parameter initialization strategies and found that CNN outperformed ViT when the data volume was small, which was attributed to the lack of inductive bias in ViT. While using the ViT model pretrained on ImageNet, the performance is comparable to CNN. If self-supervised pretraining is used, ViT outperforms CNN. They finally concluded that in medical imaging, it is reliable to replace CNN with ViT.

Although many studies have shown that deep models such as ViT have achieved remarkable performance on CV tasks, the application of ViT still requires huge computational costs. An effective way to improve model performance is to use larger datasets and increase the size of the model. Brown et al. [33] built a transformer-based GPT-3 model with 175 billion parameters, which is 10 times more than the previous largest nonsparse language model, and achieved strong performance on several NLP datasets. Zhai et al. [34] trained a ViT model with a parameter size of 2 billion, which achieved a record-breaking 90.45% on ImageNet. Applying ViT models generally requires pretraining on large datasets and then fine-tuning for (smaller) downstream tasks. Whereas large-scale training implies expensive computing power requirements, so reducing computing power while maintaining the model performance unchanged is a meaningful research direction. For the classical ViT model, the dimension size of each Transformer Encoder input and output is constant. Therefore, some researches tried to reduce the amount of transmitted data between Transformer Encoders. Pyramid ViT proposed by Wang et al. [35] constructs a sequence of Transformer Encoders, whose patch scales are reduced layer by layer, and introduces a Spacial Reduction Attention Layer before the attention module inside each encoder, which greatly reduces the computational complexity of ViT. Jaegle et al. [36] proposed the Perceiver to perform the attention mechanism in a latent space, whose size is usually smaller than the input and output, and implements the decoupling of three links of reading-processing-output, making it adaptable to inputs and outputs of different scales. Ryoo et al. [37] established a series of learned tokenizer functions, each of which converts the input image into a vector in a spacial attention calculation, thus, a set of adaptively changing informative combinations containing the pixels or spatial locations of the original image is constructed and the TokenLearner is implemented and inserted between two transformer encoders, so that the inputs of the subsequent encoders are that set of vectors instead of original patches, which greatly reduced the input size of the subsequent encoders. Meanwhile, Riquelme et al. [38] proposed Vision Mixture of Experts, a sparse version of ViT that can achieve higher performance at roughly the same computational cost, which shows that not every patch segmented off from the original image are necessary. On this basis, Renggli et al. [16] proposed Patch Merger, which amalgamates the features between different tokens in a concise way, reduces the absolute number of patches in the calculation process, and takes the reduced patch sequence as the input to the subsequent transformer encoders, thereby reducing the computational effort. This study significantly reduces the computational cost of ViT and improves the computational speed at different model sizes while maintaining the ViT performance nearly unchanged. Although Patch Merger technique shows advantages as above, the classification performance may be degraded when it is applied to medical image datasets. The reason may be that some patches containing important information may experience information loss during the conversion process. Especially for medical images, a large number of image patches may have high content similarity, while the lesion sites that play an important role in diagnosis may be relatively small, making it difficult to map the information contained in these patches to the output patches. Therefore, it is a meaningful research topic to avoid the risk of information loss brought by Patch Merger technique so that it can be more easily applied to medical imaging scenarios.

## 3. Methods

This study proposes Patch Fuser, a multisemantic level patch merger technique. It accepts enhanced training images and outputs fusioned features, which are used to perform the training of MP-ViT. Based on the self-attention mechanism of ViT, this model takes advantage of the feature dimension reduction of Patch Merger in a simple and fast way and enables the intermediate information of the Patch Merger operation to participate in the final classification. It reduces the risk of information loss that may occur in Patch Merger and further reduces the computational cost of ViT, which can promote the application of ViT in medical imaging scenarios.

The overall establishing and using pipeline of MP-ViT is described as Figure 1.

### 3.1. Transformer

The Transformer model [21] has now become one of the most popular models in the field of NLP and is widely used in the field of machine translation and achieves better performance than traditional models such as recurrent neural network (RNN) and CNN while requiring fewer computational resources. It is based on a self-attention mechanism that improves parallelization and reduces the computational difficulty of learning the similarity between distant locations to a constant level.

#### 3.1.1. Architecture

The Transformer model is based on an encoder-decoder structure. The encoder maps the input sequence *x* = (*x*_1_, ⋯, *x*_*n*_) into the sequence *z* = (*z*_1_, ⋯, *z*_*n*_). Then, an autoregressive decoder [39] generates a symbolic output sequence of the elements (*y*_1_, ⋯, *y*_*n*_). Each time the next output is generated, the previous output is transmitted to the decoder as part of the input.

The encoder-decoder structure of the Transformer model is shown in Figure 2.

*(1) Encoder*. The encoder is composed of *N* identical blocks. The first block accepts the embedded input, and the input of each subsequent block is the output of the previous block. Each block has 2 residual sublayers inside.

The first residual sublayer passes the embedded input to a multihead self-attention model, and the output of this model is summed with the input (i.e., residual structure). Then, layer normalization is performed to obtain the output of the first residual sublayer. The second residual sublayer receives the output of the first residual sublayer and then obtains the output through a simple position-wise fully-connected feedforward network. The output is also summed with its input and layer normalized to obtain the output of the second residual sublayer.

*(2) Decoder*. The structure of the decoder is similar to the encoder. It is also made up of *N* identical blocks stacked on top of each other. The decoder inserts another sublayer between the 2 residual sublayers of the encoder, which receives the multihead self-attention of the encoder output. Each sublayer is a residual structure, and the output is summed with the input and then the layer normalization is performed.

The self-attention model in the decoder stack structure is masked, i.e., it only receives the known outputs of positions smaller than *i* as input when calculating the self-attention of position *i*.

#### 3.1.2. Self-Attention Mechanism

Attention is used to describe the assigned weights of multiple elements of an input sequence, and it reflects the difference in influence of different input elements on the result. The attention function is used to map a query and a key-value pair to an output, where the query, key, value, and output are all vectors. This output is a weighted sum of the inputs, where the weight assigned to each value is the attention score which is computed from the similarity function of the query to the corresponding key.

The Transformer model takes a multihead scaled dot-product attention calculation method with the structure shown in Figure 3.

*(1) Scaled Dot-Product Attention*. The input of the model is a query, a key of length *d*_*k*_, and a value of length *d*_*v*_. The dot product of query and key is calculated first, and the result is divided by $\sqrt{d_{k}}$, then, the softmax function is applied to compute the weight of the result and then multiplied by the value. In the actual calculation, the vectors of query, key, and value are each combined into matrices *Q*, *K*, and *V*. The formula is listed as below:

(1) $$\begin{array}{c} \text{Attention}\left(Q,K,V\right)=\text{softmax}\left(\frac{QK^{T}}{\sqrt{d_{k}}}\right)V. \end{array}$$

When *d*_*k*_ is relatively large, the result of dot product after softmax calculation will be more biased towards the region with very small gradient [40], so it is divided by $\sqrt{d_{k}}$.

*(2) Multiheaded Self-Attentiveness*. To allow the model to learn information from different representation subspaces at different locations, a multihead self-attention mechanism is used. This mechanism projects query, key, and value with different, learned liner projection layers for *h* times, obtaining *h* smaller matrices of *Q*, *K*, and *V* with dimensions *dk*, *dk*, and *dv*. After *h*Attention(*Q*, *K*, *V*)s are generated, they are concatenated and the final Attention(*Q*, *K*, *V*) is obtained. The formula is as follows:

(2) $$\begin{array}{c} \text{MultiHead}\left(Q,K,V\right)=\text{Concat}\left(\text{hea}{\text{d}}_{1},\cdots ,\text{hea}{\text{d}}_{h}\right)W^{O}, \end{array}$$

where head_*i*_ = Attention(*QW*_*i*_^*Q*^, *KW*_*i*_^*K*^, *VW*_*i*_^*V*^).

And the linear projection layers are matrices of parameters:

(3) $$\begin{array}{c} W_{i}^{Q}\in {\mathbb{R}}^{d_{\text{model}}\times d_{k}},W_{i}^{K}\in {\mathbb{R}}^{d_{\text{model}}\times d_{k}}, \end{array}$$

(4) $$\begin{array}{c} W_{i}^{V}\in {\mathbb{R}}^{d_{\text{model}}\times d_{v}},W_{i}^{O}\in {\mathbb{R}}^{hd_{v}\times d_{\text{model}}}. \end{array}$$

There are 3 self-attention structures in the Transformer model. The self-attention model from encoder gets its query, key, and value from the same place, i.e., the output of the previous encoder. The masked self-attention model from decoder receives the decoder's output as input in an autoregressive approach, and the information to the right of current position will be masked (implemented by setting the input to −∞ to mask the input that should be masked). The self-attention model in the encoder-decoder layer receives the key and value from encoder and the query from masked self-attention model. This structure allows each position in the decoder to focus on all positions in the input sequence. This simulates the typical encoder-decoder attention mechanism in the seq2seq model, as in [41–43].

#### 3.1.3. Position Encoding

The self-attention mechanism calculates the weight distribution between each individual elements of a sequence regardless of the sequence order. Therefore, in order for the model to take advantage of the sequence's order, the transformer model adds position encoding information to the inputs of the encoder and decoder.

The position encoding has the dimensionality *d*_model_ which is the same as the input word embedding vector, and the result obtained by summing the position encoding and the word embedding vector is passed to the encoder and decoder as input. There are many approaches to generate position encoding including the learned way and the fixed way [42]. The Transformer model uses sine and cosine functions of different frequencies as position encoding.

(5) $$\begin{array}{c} \text{P}{\text{E}}_{\left(pos,2i\right)}=\sin\left(\frac{pos}{10000^{2i/d_{\text{model}}}}\right), \end{array}$$

(6) $$\begin{array}{c} \text{P}{\text{E}}_{\left(pos,2i+1\right)}=\cos\left(\frac{pos}{10000^{2i/d_{\text{model}}}}\right), \end{array}$$

where *pos* is the position and *i* is the dimension. For each element of the input sequence, the formula generates a vector of length *d*_model_, which uses a sine function for the even bits and a cosine function for the odd bits, so that each bit of the position-encoded vector corresponds to a sine wave and the wavelength forms a geometric progression from 2*π* to 10000 × 2*π*. For any fixed offset *k*, PE_*pos*+*k*_ can be expressed as a linear function of PE_*pos*_.

#### 3.1.4. Position-Wise Feed-Forward Networks

The self-attention sublayer output results of the encoder and decoder are passed to a position-wise feedforward neural network, which is a simple fully connected layer structure that is applied to each position separately and whose structure is identical but with different parameters. It consists of two linear transformations with a ReLU activation in between.

(7) $$\begin{array}{c} \text{FFN}\left(x\right)=\max\left(0,xW_{1}+b_{1}\right)W_{2}+b_{2}, \end{array}$$

where FFN is feed-forward networks.

#### 3.1.5. Normalizations

*(1) Internal Covariate Shift and Normalizations*. In statistics-based machine learning theory, there is a basic assumption that the source space and target space should meet the requirement of independent and identical distribution. In deep neural network, the parameters' update in each layer will lead to the change of the input data distribution of the upper layer, and through the superposition of layers, the lower space and the upper space will satisfy the assumption of “independent and identical distribution” less and less. This makes the training process difficult to converge and generates gradient explosion, gradient disappearance, overfitting, and other problems. This is the phenomenon of internal covariate shift. To solve this problem, a learnable, parameterized network layer can be introduced before or after each network layer to perform normalization.

Suppose a set of input vectors are *X* = {*x*_1_, *x*_2_, ⋯, *x*_*d*_}. Take the normalizing transformation on it so that it follows a normal distribution:

(8) $$\begin{array}{c} {\text{X}}_{\mathrm{norm}}=\frac{x-\mu }{\sigma }, \end{array}$$

where *μ* is the mean of the original data sample and *σ* is the variance. After another reshift and rescale performed, there will be a transformed input vector:

(9) $$\begin{array}{c} X_{\text{final}}=g*{\text{X}}_{\mathrm{norm}}+b, \end{array}$$

where *g* and *b* are the parameters to be learned.

*(2) Batch Normalization (BN)*. It selects a part of the samples and as a mini-batch and then normalizes a feature of all samples in the same mini-batch on a single neuron unit:

(10) $$\begin{array}{c} \mu_{i}=\frac{1}{M}\sum x_{i},\sigma_{i}=\sqrt{\frac{1}{M}\sum {\left(x_{i}-\mu_{i}\right)}^{2}+\varepsilon }, \end{array}$$

where *M* is the number of samples in the mini-batch.

BN normalizes each dimension *x*_*i*_ independently, so the ideal BN requires that the statistic quantity of each mini-batch is an approximate estimation of the overall statistic quantity, or each mini-batch should be approximately identically distributed with each other and with the overall data. It is suitable for scenarios where the mini-batch is relatively large and the data distribution is relatively similar to each other. However, if the mini-batch size is small, or the network structure is dynamic (e.g., RNN), or the length of the input and output sequences of each layer is not consistent, the BN results may be poor.

*(3) Layer Normalization (LN) [44]*. Its formula is similar to BN, but the axis of the statistics is different:

(11) $$\begin{array}{c} \mu^{l}=\frac{1}{H}\sum_{i=1}^{n}a_{i}^{l},\sigma^{l}=\sqrt{\frac{1}{H}\sum_{i=1}^{n}{\left(a_{i}^{l}-\mu^{l}\right)}^{2}}, \end{array}$$

where *H* is the number of neurons in that layer of the neural network.

The LN performs normalization to all features of the same sample, and all neurons in that layer share this normalized mean and standard deviation. Therefore, LN is not affected by the data distribution in the mini-batch, regardless of the mini-batch size or the number of samples in the input sequence. It is suitable for scenarios such as small mini-batch, dynamic network structure, and RNN, and it is used in Transformer model.

### 3.2. Vision Transformer

Transformer works well in NLP domain. In 2020, Dosovitskiy et al. [13] applied Transformer from NLP to CV with the least change and built Vision Transformer (ViT) model to verify the effectiveness of Transformer use in CV. Experiments show that the performance of ViT is comparable to the best CNN on large datasets and consumes less computational resources (it is a little lower than CNN on medium datasets, which is attributed to the lack of inductive bias that CNNs have).

#### 3.2.1. The Difficulty of Taking Usage of Transformer in CV

Transformer is based on the self-attention mechanism, and the computational complexity is *O*(*n*^2^), in which *n* means the sequence length. The image information is the input sequence. If a 2D image is directly spread by pixel, a 224 × 224 image can be expanded to a sequence of 50,176 pixel points, which is too large to be computed under existing hardware conditions.

#### 3.2.2. The Solution

To reduce the computational effort, the size of input data should be controlled. Since it is too long when the image is expanded by pixel, if a large image is divided into several patches, each is transferred to the Transformer model as input, the sequence length can be reduced. E.g., for a 224 × 224 image, we divide it into 14 × 14 = 196 small patches, the sequence length 196 is acceptable, and the resolution of each patch is 16 × 16 = 256.

#### 3.2.3. Model Architecture

The ViT model nearly keeps the Transformer structure the same and utilizes the encoder part, and the input data is processed by encoder and then directly used to classification without the decoder part. Its structure is shown in Figure 4.

*(1) Data Preprocessing*. First, the image is divided into several small patches, and each patch is transformed into a patch embedding by the linear projection layer, so that an image is transformed into a sequence. Then, similar to the Transformer model, the position embedding of each patch and the features of the image is added together to form a sequence of length *n*, here, *n* = *H*∗*W*/*n*_patch_∗*C*, where *H*∗*W* is the image resolution, *n*_patch_ is the number of nuggets, and *C* is the number of channels.

Similar to BERT [22], patches are linearly projected, and a classification token is appended with position embedding (fixed to 0) and transmitted to the Transformer encoder as input. This classification token is a learnable embedding result for the final classification usage.

*(2) ViT Encoder*. Similar to Transformer, the encoder consists of *L* blocks, and each block has two residual sublayers which are used to perform the calculation of multihead self-attention mechanism and the MLP. The main difference is that in Transformer, the data is computed first before layer normalization, while the ViT model performs layer normalization first and then performs the computation of multihead self-attention or MLP. The MLP has two hidden layers and uses the GELU nonlinear activation function. The computation process is shown in the following equation:

(12) $$\begin{array}{c} z_{0}=\left[x_{\text{class}};x_{p}^{1}E;x_{p}^{2}E;\cdots ;x_{p}^{N}E\right]+E_{pos},E\in {\mathbb{R}}^{\left(P^{2}\cdot C\right)\times d},E_{pos}\in {\mathbb{R}}^{\left(N+1\right)\times D}, \end{array}$$

(13) $$\begin{array}{c} z_{l}^{\prime }=\text{MSA}\left(\text{LN}\left(z_{l}-1\right)\right)+z_{l-1},l=1,2,\cdots ,L, \end{array}$$

(14) $$\begin{array}{c} z_{l}=\text{MLP}\left(\text{LN}\left(z_{l}^{\prime }\right)\right)+z_{l}^{\prime },l=1,2,\cdots ,L, \end{array}$$

(15) $$\begin{array}{c} y=\text{LN}\left(z_{L}^{0}\right), \end{array}$$

where *x*_class_ is the classification token, *E* means input embedding, *E*_*pos*_ means the position embedding, MSA is multiheaded self-attention model, MLP is the perceptron, LN is layer normalization, and *y* is the image representation computed from the output result of the last ViT encoder.

*(3) Classification Head*. After the computation in ViT encoder finished, the output vector corresponding to the classification token is used as the basis for classification. It is passed to the classification head for classification. The classification head is an MLP with a hidden layer in pretraining and a simple linear layer in fine-tuning.

*(4) Position Embedding*. The position encoding in Transformer encodes position information using sine and cosine functions. Unlike this, ViT uses a learnable one-dimensional position embedding.

#### 3.2.4. Model Application Method

After the initial ViT model is obtained by pretraining on a large dataset, it can be fine-tuned for smaller downstream task datasets. In fine-tuning, the classification head of the pretrained ViT is removed and replaced by a zero-initialized *D* × *K* feed-forward layer, where *K* is the number of classifications in the target dataset. When the resolution of the target dataset gets higher, the resolution of each patch is maintained, so that more image patches are obtained, and therefore, the original position embedding information is meaningless. Thus, it needs to perform two-dimensional interpolation of the pretrained positional embeddings according to their positions in the original images.

#### 3.2.5. Why ViT on Medical Images

Medical X-ray images are characterized by the fact that the images are usually grayscale distributions with similar styles in most areas. The key of classification is to find out the structure of the lesion site and to identify the boundary between the lesion and the surrounding tissue. The main difference between normal images and lesion images lies in the lesion part, which may be relatively small.

These features make it possible for ViT to achieve better results on medical X-ray images. ViT divides the image into small patches, and its self-attention mechanism provides the following advantages:

1. It is able to capture long-distance dependencies and learn efficient feature representations [45] to model the relationships between spatially distant patches
2. It computes attention scores among image patches and uses them as weights to model the input adaptively, determining the individual image patch importance relative to other patches, thus, capturing the relationship between two image patch and preventing the model from influences of a large number of similar patch on the classification
3. It learns the correspondence between the global context and the key patches that distinguish normal and diseased tissues, thus, preventing the model from misclassification

### 3.3. Label Smoothing

Label smoothing is a technology to prevent neural networks from overconfidence that leads to overfitting and has been widely used by advanced models in many fields. It has been shown that label smoothing can improve the generalization ability of the model and help to improve the performance [46, 47].

In classification tasks, the category label *y*_*i*_ of training data is generally represented by 0 or 1 in one-hot encoding as below:

(16) $$\begin{array}{c} y_{i}=\left\{\begin{array}{cc} 1, & i=\text{target},\\ 0, & i\neq \text{target}. \end{array}\right. \end{array}$$

The cross-entropy loss function is

(17) $$\begin{array}{c} H\left(y,p\right)=-\overset{K}{\underset{i}{\sum }}y_{i}\log P_{i}, \end{array}$$

where *p*_*i*_ is the value of the logit vector *z*_*i*_'s function calculated by softmax, and *z*_*i*_ is generated from the penultimate layer vector outputs of the model:

(18) $$\begin{array}{c} p_{i}=\frac{\exp\left(z_{i}\right)}{\sigma_{j}^{K}\exp\left(z_{j}\right)}. \end{array}$$

#### 3.3.1. The 0-1 Labeling Problem

In the learning process of neural networks, the “0 or 1” label drives the model to learn in the direction that the probability of the target category tends to 1, and the probability of non-target category tends to 0. This makes the final predicted logits vector *z*_*i*_'s value of the target category tend to infinity (so that the probability distribution of the softmax output is more extreme and tends to be more bipolar), resulting in the model's unadaptiveness and overconfidence in its predictions. The training data is insufficient to cover all cases, and with some labeled data not necessarily accurate, this can easily lead to overfitting of the network and poor generalization ability.

#### 3.3.2. Label Smoothing

It takes label vectors instead of one-hot encoded 0 or 1 labels $\hat{y}$:

(19) $$\begin{array}{c} {\hat{y}}_{i}=y_{\text{hot}}\left(1-\alpha \right)+\frac{\alpha }{K}, \end{array}$$

where *K* is the total number of classifications and *α* is a tunable hyperparameter (e.g., 0.1), i.e.,

(20) $$\begin{array}{c} {\hat{y}}_{i}=\left\{\begin{array}{cc} 1-\alpha , & i=\text{target},\\ \alpha /K, & i\neq \text{target}. \end{array}\right. \end{array}$$

The cross-entropy loss function is also changed accordingly as follows:

(21) $$\begin{array}{c} \text{Loss}=-\overset{K}{\underset{i=1}{\sum }}p_{i}\log q_{i}\Rightarrow \text{Los}{\text{s}}_{i}=\left\{\begin{array}{cc} \left(1-\alpha \right)*\text{Loss}, & ,\text{if}\left(i=y\right),\\ \alpha *\text{Loss}, & ,\text{if}\left(i\neq y\right). \end{array}\right. \end{array}$$

This reduces the output values difference between the predicted positive and negative samples, prevents the model from being overconfident on the correct labels, and makes the clusters of different classifications more compact. It also increases the interclass distance and decreases the intraclass distance, thus, avoiding overfitting and improving the generalization ability of the model.

### 3.4. Patch Merger

Compared to traditional networks like CNNs, ViT has reduced the computational cost but still require a large computational effort. In NLP, the Sparse Mixture of Experts (MoE) [48] model extends the number of model parameters to the trillion level, while for each input sample, only a small subset of the sparse parameters is applied to compute. This idea of conditional computation was extended to CV by Riquelme et al. [38]. They established the Vision Mixture of Experts (V-MoE) model, which proposes the Batch Prioritized Routing (BPR) algorithm to prioritize each token (a token is a patch input to encoder) and discard some least important tokens. Based on that, Patch Merger proposed by Renggli et al. [16] significantly reduces the number of image patches required for classification at the early stages of the ViT operation with minimal additional computational cost, while keeping performance essentially constant.

#### 3.4.1. Model Architecture

Patch Merger is applied between 2 transformer encoders. It takes an input of any dimensionality and produces an output of the specified dimensionality (which is generally smaller than the input dimensionality). The subsequent ViT encoders receive the input of the new (smaller) dimensionality.

The architecture of Patch Merger is shown in Figure 5.

Patch Merger is a learned *D* × *M* matrix *W* (where *M* is the number of output patches and *D* is the number of embedding dimensionality). After layer normalization, the input matrix *X* ∈ ℝ^*N*×*D*^ (i.e., *N* input patches, each with embedding dimension *D*) is multiplied with *W*. The result is transposed and then normalized by softmax and multiplied with matrix *X* to obtain the score-weighting matrix *X* ∈ ℝ^*N*×*D*^ of all output patches:

(22) $$\begin{array}{c} Y=\text{softmax}\left({\left(XW\right)}^{T}\right)X=\text{softmax}\left(W^{T}X^{T}\right)X. \end{array}$$

This formula is similar to the self-attention formula of Transformer:

(23) $$\begin{array}{c} \text{Attention}\left(Q,K,V\right)=\text{softmax}\left(QK^{T}\right)V. \end{array}$$

This is equivalent to simply learning a fixed set of queries for each input patch, using the input patch as key and value.

Patch Merger is located between two neighboring ViT encoders.

#### 3.4.2. Why Patch Merger Works and the Risk

The processing of Patch Merger is to map the input features to the high-level semantic space and then take dimensionality reduction in the high-level space to reduce the number of features while preserving the original semantic features as much as possible, thus, reducing the computational effort and maintaining the basic model performance at the same time. Each output patch contains the weighted information of all input patches, and the weights (i.e., matrix elements of patch merger) indicate the influence degree of each input patch on the output patch.

Input patches with high similarity and low impact on the classification are similarly routed, i.e., they are eventually contributed or output to the same subset of output patches. This mechanism is useful, for example, in object-centric images, where the semantics of repeated and similar background patches are compressed into the same output patches, thus, reducing the redundant computation amount in subsequent ViT encoders. The input patches, which play a key role in classification, affect the other output patches more. This may be an advantageous factor for applying patch merger to medical images, because some medical images (e.g., normal and pneumonia chest images in this paper) may have most patches similar to each other, and the lesions account for a small percentage, so these output patches containing more semantic information of lesions are more likely to be influenced by the input patches of lesions. This may be the reason why Patch Merger can work.

In addition, Patch Merger has some interesting features. For example, the way input patch is assigned to output patch is independent of the original position of input patch. What is more, we can freely change the number of input patches while keeping the learned parameters unchanged.

The main risk that may arise from applying patch merger is the loss of semantic information. Some input patches contain diverse information, where features that have a significant impact on classification may not be obvious. After mapping them to the high-level semantic space for dimensionality reduction and then process them in subsequent multiple ViT encoder, these features may decay to a very weak and unnoticeable level (especially when there are too many ViT encoders), which causes semantic loss. Especially for some medical images, it is possible that semantic information is lost when it is not obvious to determine whether the image indicates a lesion for a certain disease or not.

#### 3.4.3. Patch Merger Design Choice

Because Patch Merger reduces the number of input patches for the subsequent ViT encoder, it also reduces the computational cost. If Patch Merger is added too early, the computation effort can be reduced greatly, but the performance of the model may not be ideal. If it is added too late, however, there will be little effect on the computation effort.

The study of Renggli et al. [16] chose to add Patch Merger blocks in the middle of two half parts of the original network (ViT or V-MoE). For example, if the original network has 8, 12, 24, and 32 ViT encoders, Patch Merger is added after the 4th, 6th, 12th, and 16th ViT encoder. The number of output patches of Patch Merger is always set to 8. Experiments show that this design greatly reduces the computational cost of the second half of the original network and maintains comparable performance of the original model.

### 3.5. Patch Fuser

Based on Patch Merger, we propose the Patch Fuser for ViT in order to reduce the risk of semantic information loss while taking advantage of the reduced computational cost introduced by the application of Patch Merger. Considering that the risk is mainly brought by the Patch Merger's output patches being processed by subsequent ViT encoders, and the Patch Merger's output patches can be regarded as the intermediate result which still contain the semantic information that may get weaker and weaker in the subsequent processing and eventually be lost, we expect to utilize these intermediate results and let them participate in the final classification, thus, avoiding semantic loss.

The architecture of Patch Fuser is described in Figure 6.

The model contains L ViT encoders (numbered 1 to L, respectively), and a Patch Merger is added after each of the two trilaterals (i.e., the *L*/3th and the 2*L*/3th encoder). The output patches from these two Patch Mergers are not only processed further by the subsequent ViT encoders but also fused with the output of the last encoder to obtain the fusioned features. These features contain intermediate information for data processing.

Assuming that the original input patches consist of an *N* × *D* matrix, where *N* is the number of patches and *D* is the size of the hidden dimension (that is, the dimension size of the embedding of each patch), the input and output of each ViT encoder are both *N* × *D* matrix. After processed by the first Patch Merger, the result is changed to an *M* × *D* matrix, which is the 1st intermediate result, where the hyperparameter *M* is the number of output patches of the Patch Merger. The input of each subsequent ViT encoder and the 2nd Patch Merger is MÃ—D matrices. The second Patch Merger outputs the 2nd intermediate result. Finally, the two intermediate results are concatenated with the output of the last ViT encoder to form an *M* × *D* × 3 tensor, and then the tensor is fused by a one-dimensional convolution with kernel size = 1 to produce an *M* × *D* matrix as the fusioned features.

The main consideration of this design is that the intermediate results of output patches of Patch Merger contain semantic information that may be decayed, so the intermediate results are kept and allowed to fuse directly with the output results of the last ViT encoder, thus, avoiding the loss of semantic information. It is also inspired by ResNet: if the whole model is delimited into 3 modules by Patch Merger, it is equivalent to let the input of the first two modules enter the next operation step together with the output of the last module. This helps to preserve as much semantic information as possible and allows a smoother backward and forward propagation of the model.

The MP-ViT contains our Patch Fuser. The fusioned features generated by Patch Fuser are fed to the final MLP Head for classification along with the smoothed labels, and the output is the final classification result. Thus, the training process of MP-ViT is completed.

## 4. Experiments

In this section, through experiments, we demonstrated that the MP-ViT proposed by us with application of label smoothing and image enhancement techniques results in better performance compared to baseline (ResNet50), ViT, ViT + Patch Merger, etc.

### 4.1. Dataset

The dataset used in this study was presented by Kermany et al. in 2018 [49], and it contains 5,232 chest X-ray images from children under 5 years of age. Among them, there are 1,349 normal chest samples and 3,883 samples identified as pneumonia, which are used as the training set. The test set consists of another 624 images from other patients, including 234 normal samples and 390 pneumonia samples. The negative and positive categories in the training and test sets are 1 : 2.878 and 1 : 1.667, respectively.

### 4.2. Image Enhancement

X-ray images are obtained by producing pixels of different brightness according to the absorption values of the individual voxels. For example, in a chest radiograph, X-rays pass through the lungs with little attenuation, while they are strongly absorbed through the thoracic spine, thus, they show different brightness on different pixels of the image. The disease diagnosis relies on the doctors' findings of very fine details in the image, such as lesions of lung nodule. And image enhancement can make some details more visible, helping doctors improve diagnosis and making CAD more accurate. Unsharp Masking (UM), one of the image enhancement methods widely used in medical imaging, sharpens the mid and high frequency components of an image and preserves the low frequency components, so that details with weaker contrast are more visible while keeping the intensity of the large areas of the image [50]. To enhance the image quality and allow the computer to recognize pneumonia more easily, this study applied UM to all images and compared them. Radius is used to indicate the blurring intensity to 1, and the amount is used to indicate the intensity of the edges (how much dark or light it will be) to 15. The comparison between the UM-enhanced images and the original images is shown in Figure 7.

### 4.3. Training Details

We uploaded the original images as the model input to cloud environment, on which we first trained with ResNet50 as a baseline for comparison. Then ViT model, ViT + Patch Merger model, and MP-ViT model were trained with the same dataset. Finally, the MP-ViT proposed by us was trained again with the UM-enhanced images as input and the label smoothing technique was introduced in order to compare the performance of the 5 different models as well as the image enhancement and label smoothing.

#### 4.3.1. Hardware

The training process took place in the cloud environment, and the cloud server hardware configuration is listed below. The CPU is 7-core Intel (R) Xeon (R) CPU E5-2680 v4 @ 2.40 GHz, while the GPUs are 2 RTX 3090 (24 GB) graphic cards, and the RAM is 32 GB.

#### 4.3.2. Training Configs

The Python version used for training is 3.8, the machine learning framework is PyTorch 1.10.0, and the CUDA version is 11.3. The maximum number of training epoch for all models is 200. Learning rate is set to 0.00001, and the epsilon value for label smoothing is 0.01 in the final model.

### 4.4. Results

We performed classification on the test set with the models obtained from training and compared the performance of these models using statistical metrics such as accuracy, precision, recall, and *F*1-score, which are widely used to measure the performance of classifiers and also showed the variation of the loss curves.

#### 4.4.1. Accuracy

For a classification task, each classification prediction may be one of the following four results: (1) it is predicted as positive and the result is positive, i.e., true positive (TP); (2) it is predicted as negative and the result is negative, i.e., true negative (TN); (3) it is predicted as positive but the result is negative, i.e., false positive (FP), which is called statistical type I error; (4) it is predicted as negative but the result is positive, i.e., false negative (FN), which is called statistical type II error. Among them, TP and TN are predicted correctly, and FP and FN are predicted wrongly. The accuracy rate is the ratio of the number of correct predictions to the total number of predictions, and the formula is as follows:

(24) $$\begin{array}{c} \text{Accuracy}=\frac{\text{TP}+\text{TN}}{\text{TP}+\text{TN}+\text{FP}+\text{FN}}. \end{array}$$

#### 4.4.2. Other Statistical Metrics

In addition to accuracy, other metrics are also used to evaluate the performance of classifiers. The most common ones are precision, recall, and *F*1-score.

Precision refers to the ratio of the number of samples that are actually positive to the number of samples that are predicted to be positive. A high precision indicates that the classifier predicts a positive result with high reliability, but there may be actual positive samples that have been missed. The formula is as follows:

(25) $$\begin{array}{c} \text{Precision}=\frac{\text{TP}}{\text{TP}+\text{FP}}. \end{array}$$

Recall refers to the ratio of the number of samples predicted to be positive to the total number of samples that is actually positive. A high recall means that the classifier will miss as few positive samples as possible, but samples that are actually negative may also be predicted to be positive. The formula is as follows:

(26) $$\begin{array}{c} \text{Recall}=\frac{\text{TP}}{\text{TP}+\text{FN}}, \end{array}$$

As can be seen, precision and recall are sometimes contradictory, and raising one may lower the other. The *F*-measure is a comprehensive indicator, which is the weighted summed average of precision and recall, and its calculation formula is as follows:

(27) $$\begin{array}{c} F=\frac{\left(\alpha^{2}+1\right)*\text{precision}*\text{recall}}{\alpha^{2}*\left(\text{precision}+\text{recall}\right)}, \end{array}$$

where *α* is the importance weighted index of recall relative to precision, and depending on its value, the *F*-measure is a different *F*-score. For example, the *F*2 score gives 2 times the importance of recall compared to the *F*1 score. The commonly used *F*-measure is the *F*1-score, which is calculated as follows:

(28) $$\begin{array}{c} F1=\frac{2*\text{precision}*\text{recall}}{\text{precision}+\text{recall}}. \end{array}$$

#### 4.4.3. Model Performance Comparison

In general, the dataset of this study did not suffer from severe class imbalance, and the metrics showed consistent trends among the models. To simply compare the performance of these models, we did not use any special trick to train the models. The detailed comparison of several models is shown in Tables 1 and 2, where M1, M2, and M3 mean baseline, ViT, and Patch Merger, respectively.

The baseline (M1) accuracy is 86.86% with an *F*1-score of 85.14%, which is an ideal result. Its initial training and testing losses are around 0.7, and their values changed smoothly with epoch increasing, and they finally converge to around 0.27 and 0.35, respectively. Its loss curve is listed as Figure 8.

ViT (M2) had the lowest metrics with an accuracy of 77.72% and an *F*1-score of 74.46%, which is significantly lower than the baseline. The training and testing losses of ViT experienced a significant increase after the first 10 or so epochs of rapid reduction and then continued to decrease. The final training and testing losses of ViT (0.42 and 0.5) are significantly higher than other models. As described in Methods, the less ideal performance of ViT directly trained on small datasets may be attributed to the lack of priori inductive bias compared to CNN. The loss curve is listed in Figure 9.

The accuracy of Patch Merger (M3) reaches 88.94%, and the *F*1-score is 87.85%, which is slightly higher than the baseline. The change trend of its loss curves is similar to that of ViT, which experienced a process of a rapid decrease and then an increase and a decrease again. The final training and test losses are 0.23 and 0.38, respectively. As can be seen, Patch Merger can sometimes display better performance than ViT, which may be brought by the feature amalgamation performed by Patch Merger: the redundant information is discarded, and the more expressive part is retained. Its loss curve variation is shown in Figure 10.

The accuracy of our proposed MP-ViT is improved to 89.74%, and the *F*1-score is also improved to 88.67%. The loss curve tends to be smooth again with less oscillation, and the training and testing losses eventually drop to 0.24 and 0.3, which was better than the previous model. This may be attributed to MP-ViT's ability to learn across semantic levels and to model from local to global. The change of its loss curve is shown in Figure 11.

Finally, with the application of image enhancement and label smoothing technology to our MP-ViT model, the accuracy is improved to 91.19%, and *F*1-score is also improved to 90.34%. The training and testing loss values are further reduced to 0.23 and 0.29, respectively. It is shown that the image enhancement and label smoothing are indeed beneficial to improve the model performance. The loss curve of the final model is demonstrated in Figure 12.

## 5. Conclusion and Future Work

In this study, we propose MP-ViT to perform classification on medical images and compare it with ResNet50 (baseline), ViT, and Patch Merger and also tried to apply label smoothing and image enhancement technology to further improve the model performance. Without using other tricks, the accuracy and *F*1-score of the baseline are 0.868590 and 0.851442, respectively, while those of our model are 0.911859 and 0.903365, respectively. Our model achieved better performance than the baseline, ViT, and Patch Merger. Meanwhile, label smoothing and image enhancement technologies also achieved better results.

Our proposed model attempts to utilize the intermediate results of ViT and Patch Merger to retain information from the transformation process of the high-level semantic space to participate in the final classification. This can not only take advantage of the self-attention mechanism of ViT but can also maintain the advantage of low computational cost of Patch Merger and also avoid the risk of semantic information loss. The application of label smoothing and image enhancement techniques further improves the model performance. For medical imaging, these advantages are especially useful, because most of the areas in medical images may not be useful for disease diagnosis and have high similarity, while the actually useful parts may be small and unclear, so the semantic intermediate information of the spatial transformation preserved can be a key point in maintaining model performance. In addition, the production cost of medical imaging datasets is high because it requires a lot of expert judgments. Our model can show high performance on smaller medical imaging datasets without pretraining, which demonstrates that our model is not expensive. These advantages can work well for CAD of medical images.

Although our model has achieved better results than ViT and Patch Merger, there are still some shortcomings listed as below:

1. The number of patches output from each Patch Fuser is currently set as a hyperparameter, and there is no adaptive mechanism of setting patch number
2. There is no exploration on whether the number of output patches from Patch Fusers at different semantic level should be set to be the same
3. Further experiments performed on more and larger datasets are needed

In future research work, we will search for a more reasonable mechanism for setting the number of patches and also run more experiment on larger-scale image datasets to improve our model.

## Figures and Tables

**Figure 1:** The overall establishing and using pipeline of MP-ViT Model. The raw images are input to the Patch Fuser after image enhancement and layer normalization, and then the fusioned features are obtained after model process. Those fusioned features are trained together with smoothed labels to build MP-ViT Model, and then it is used for prediction.

**Figure 2:** The model structure of Transformer.

**Figure 3:** (a) The calculation of scaled dot-product attention. (b) Structure of multihead attention calculation in parallel.

**Figure 4:** The input image is split to several patches and then linearly embedded; then, the position embedding is added to the result sequence. The sequence is fed to several Transformer encoders. An extra learnable classification token is also added into the input sequence.

**Figure 5:** (a) Overview of Patch Merger architecture and the input/output streams. It receives an input sequence of length n and produces an output sequence of length *M* (usually *M* < *n*). (b) The location of the application of Patch Merger.

**Figure 6:** Overview of Patch Fuser architecture. The output patches of each Patch Merger are saved as intermediate results that participate in the final feature fusion.

**Figure 7:** Comparison of original and UM-enhanced images. (a) is the original chest image of a normal sample and (b) is the corresponding UM-enhanced image; (c) is the original chest image of a sample diagnosed with pneumonia and (d) is the corresponding UM-enhanced image.

**Figure 8:** The loss curve change of baseline (M1).

**Figure 9:** The loss curve change of ViT (M2).

**Figure 10:** The loss curve change of Patch Merger (M3).

**Figure 11:** The loss curve change of MP-ViT.

**Figure 12:** The loss curve change of MP-ViT with image enhancement and label smoothing.

**Table 1:** Result comparison between models: accuracy.

Model	ViT	Patch merger	Patch fuser	Label smoothing	Image enhancement	Accuracy
M1	X	X	X	X	X	0.868590
M2	✓	X	X	X	X	0.777244
M3	✓	✓	X	X	X	0.889423
MP-ViT	✓	✓	✓	X	X	0.897436
Final model	✓	✓	✓	✓	✓	0.911859

**Table 2:** Result comparison between models: precision, recall, and *F*1-score center.

Model	ViT	Patch merger	Patch fuser	Label smoothing	Image enhancement	Precision	Recall	*F*1-score
M1	X	X	X	X	X	0.886129	0.835897	0.851442
M2	✓	X	X	X	X	0.779524	0.733761	0.744629
M3	✓	✓	X	X	X	0.893820	0.868803	0.878513
MP-ViT	✓	✓	✓	X	X	0.905961	0.875214	0.886710
Final model	✓	✓	✓	✓	✓	0.918173	0.893590	0.903365

## Data Availability

The data used to support the findings of this study are included within the article. All images were obtained from the Guangzhou Women and Children's Medical Center. The second version of this dataset is used, and it is licensed under the Creative Commons Attribution 4.0 International License. All data is available for downloading at this website: https://data.mendeley.com/datasets/rscbjbr9sj/2.
